The article "A novel therapeutic strategy of combined camrelizumab and apatinib for the treatment of advanced hepatocellular carcinoma" was retracted in 2024. Reasons: compromised peer review; concerns about the results or conclusions; concerns about the peer review; concerns about a third party's involvement.

# A novel therapeutic strategy of combined camrelizumab and apatinib for the treatment of advanced hepatocellular carcinoma

**DOI:** 10.3389/fonc.2023.1136366

**Published:** 2023-03-29

**Authors:** Qing Yang, Gengyu Li, Xiaoqiu Wu, Haiying Lin, Wanrui Wu, Xiangpang Xie, Yu Zhu, Wei Cai, Changsheng Shi, Shengye Zhuo

**Affiliations:** ^1^ Department of Gastroenterology, The Third Affiliated Hospital of Wenzhou Medical University, Wenzhou, Zhejiang, China; ^2^ Interventional vascular Surgery, The Third Affiliated Hospital of Wenzhou Medical University, Wenzhou, Zhejiang, China

**Keywords:** Apatinib, camrelizumab, hepatocellular carcinoma, advanced stage, tumor markers

## Abstract

**Methods:**

83 patients with hepatocellular carcinoma (HCC) admitted to the interventional oncology department were randomly divided into two groups. Apatinib and camrelizumab were administered to 42 patients in group A, whereas sorafenib was administered to 41 patients in group B for three months. The clinical efficacy was evaluated in terms of objective response rate (ORR), and disease control rate (DCR). Certain tumor markers like alpha-fetoprotein (AFP), carbohydrate antigen 199 (CA199), carcinoembryonic antigen (CEA), hypoxia-inducible factor (HIF-1), immune function T lymphocyte subsets (CD3+, CD4+, CD8+, CD4+/CD8+) were determined before and after treatment. The serum levels of vascular endothelial growth factor (VEGF), osteopontin (OPN), aspartate aminotransferase (AST), and epidermal growth factor 7 (EGF7)] were observed. The survival time between the two groups was compared, such as progression-free survival (PFS) and median survival (MS). Finally, the toxicity and side effects data were also obtained.

**Results:**

The ORR and DCR of group A were 69.05% and 88.10%, respectively, which were significantly higher (P<0.05) than group B (ORR=53.66% and DCR=70.73%). After treatment, the AFP, CA199, CEA, and HIF-1 levels of both groups decreased significantly (P<0.05), and the respective biomarker levels of group A were lower than those of group B (P<0.05). Following treatment, CD3+, CD4+, CD4+/CD8+ index in group A significantly increased (P<0.05) while CD8+ level was significantly decreased (P<0.05). Compared to group B, a significant increase was observed in group A’s CD3+, CD4+, and CD4+/CD8+ index. There were no significant changes in CD3+, CD4+, CD8+, CD4+/CD8+ indexes before and after treatment in group B (P>0.05). The serum level of VEGF, OPN, EGF-7 and AST indexes of group A&B were decreased significantly (P<0.05). Compared with group B, the VEGF, OPN, EGF7 and AST indexes of group A were significantly reduced (P<0.05). PFS and MS in group A were significantly higher than in group B (P<0.05). There was no significant difference between groups A and B in terms of toxicity and adverse effects (P>0.05).

The article "A novel therapeutic strategy of combined camrelizumab and apatinib for the treatment of advanced hepatocellular carcinoma" was retracted in 2024. Reasons: compromised peer review; concerns about the results or conclusions; concerns about the peer review; concerns about a third party's involvement.

**Conclusion:**

In treating HCC, combining apatinib and camrelizumab can reduce tumor markers, enhance the immune system and curative effect, and prolong patient survival. The underline mechanism is related to the down-regulation of VEGF, OPN and HIF-1 indexes.

## 1 Introduction

Hepatocellular carcinoma (HCC) is the most prevalent histological subtype of liver cancer, comprising 85 to 90 per cent of primary liver cancer (PLC), with a high mortality rate and ranking as the third leading cause of cancer-related death worldwide (1). The major risk factors for HCC are genetics, chronic hepatitis B, and smoking. This malignant tumor develops perniciously. When most patients are diagnosed, they are in the middle or late stages and lose the best surgery opportunity. Advanced HCC is typically treated with liver transplantation, molecular targeted therapy, radiation and chemotherapy, and immunotherapy. Liver transplantation is the most effective therapy among them. However, most patients are not transplant candidates due to tumor burden and liver function issues. Sorafenib is a novel targeted therapeutic drug that inhibits vascular endothelial growth factor and platelet-derived growth factor (PDGF) receptors, thereby inhibiting tumor progression, recurrence, and metastasis. Apatinib is a new generation of small-molecule anti-angiogenic targeted drugs that can improve liver function in patients with advanced HCC (2). Apatinib, as a small-molecule tyrosine kinase inhibitor, treats hepatocellular carcinoma mainly through targeted inhibition of tumor neovascularization, promotion of apoptosis of hepatocellular carcinoma cells, and finally inhibition of tumor progression (3). B-cellomato-2 gene (Bcl-2) plays a key role in the apoptosis-related signaling pathway of hepatoma cells. Bcl-2 can inhibit the apoptosis of hepatocellular carcinoma cells and promote the proliferation of hepatocellular carcinoma cells. In 2014, Apatinib was approved by the national Food and Drug Administration for the first time for the treatment of malignant tumors after phase III clinical trials (4). The AHELP study reported at ASCO Annual Meeting in 2020 confirmed that Apatinib, as a second-line therapy, can indeed improve the survival benefits of patients with advanced HCC (4). Apatinib also became the only targeted drug that received indications for the treatment of hepatocellular carcinoma in China that year, and was recommended as a second-line treatment for liver cancer by the CSCO guidelines in the same year (4). According to the report of the 2018 ESMO Annual meeting, the Phase 11 clinical study of carrilizumab in the treatment of advanced hepatocellular carcinoma has also achieved good results (5). All these indicated that the independent development of immunotherapy and targeted therapy drugs in advanced hepatocellular carcinoma reached a new height. According to previous studies, molecular targeted therapy or chemotherapy combined with immunotherapy can induce immunological prototypical cell death (ICD) in cancer cells more effectively and have a synergistic effect (6). Programmed cell death protein-1 (PD-1) is a key immunosuppressive molecule with potent antitumor activity in oesophagal squamous cell carcinoma, gastric cancer, non-small cell lung cancer, and liver cancer (7). Camrelizumab is a novel humanized immunoglobulin G4 (IgG4) monoclonal antibody that targets PD-1 by inhibiting its binding to programmed death ligand 1 (PD-L1), promotes the recovery of the body’s immune function and exerts an antitumor effect, thereby offering a new approach for optimizing the treatment plan for HCC.

The article "A novel therapeutic strategy of combined camrelizumab and apatinib for the treatment of advanced hepatocellular carcinoma" was retracted in 2024. Reasons: compromised peer review; concerns about the results or conclusions; concerns about the peer review; concerns about a third party's involvement.

In this study, apatinib and camrelizumab were used to treat HCC, and tumor markers, immune function, and serum indexes were observed and analyzed to evaluate the safety and efficacy of the treatment regimen quantitatively.

## 2 Materials and methods

### 2.1 General information

88 HCC patients hospitalized in the Department of Oncology from June 2019 to June 2020 were the subjects of this study. Using the random number table method, they were divided into groups A and B, with 44 cases in each group according to the 1:1 principle. Two patients in group A discontinued treatment for personal reasons, two in group B abandoned follow-up, and one was excluded for refusing laboratory testing. As indicated in **Table S1**, there were no statistically significant differences between the two groups regarding gender, disease progression, BMI, and other variables (P>0.05). The Medical Ethics Committee assessed and approved this study.

### 2.2 Case selection

#### 2.2.1 Diagnostic criteria

Imaging, serological, and pathological examinations that meet diagnostic criteria for HCC as specified in the “Guidelines for Standardized Pathological Diagnosis of Primary Liver Cancer (2015 Edition)” (8).

#### 2.2.2 Inclusion criteria

(1) Barcelona Liver Cancer Clinical Staging System (BCLC) stage: B to C; (2) Karnofsky (KPS) score >70; (3) No history of HCC-related treatment; (4) Primary ≥1 lesion with a diameter of ≥1cm; (5) Have not participated in other studies recently; (6) Patients can tolerate immune and targeted therapy; (7) The patients and their families are informed and signed the informed consent.

The article "A novel therapeutic strategy of combined camrelizumab and apatinib for the treatment of advanced hepatocellular carcinoma" was retracted in 2024. Reasons: compromised peer review; concerns about the results or conclusions; concerns about the peer review; concerns about a third party's involvement.

#### 2.2.3 Exclusion criteria

(1) Combined with other primary malignant tumors; (2) Combined with haematological or autoimmune diseases; (3)The expected survival period is less than 3 months; (4) hypertension that is poorly controlled by drugs; (5) Major organ bleeding or gastrointestinal bleeding occurred in the past 7 days; (6) Combined with mental disorders; Patients who are allergic to related ingredients, or who are prone to allergies. (7) Patients who did not meet the inclusion criteria; (8) Those who gave up treatment due to personal reasons during the treatment period; (9) Those who could not cooperate with completing relevant biochemical examinations and imaging examinations during the trial; (10) Those who had incomplete clinical data.

### 2.3 Treatment methods

After the patients were enrolled, various tests were conducted, and their physical status was comprehensively assessed. Group A was treated with apatinib (Jiangsu Hengrui Medicine Co., Ltd.; Guoyao Zhunzi H20140104; specification 0.25g) combined with camrelizumab (Jiangsu Hengrui Medicine Co., Ltd.; Guoyao Zhunzi S20190027; specification 200mg/bottle). Apatinib was orally administered 30 minutes after meals (250 mg), once a day. Camrelizumab, (200 mg), diluted with 100 ml of 0.9% sodium chloride injection, was administered intravenously every 3 times once a week if the patient is experiencing mild side effects during treatment and can tolerate it, the treatment should continue as scheduled. If there are grade 3 or higher adverse effects, such as abnormal liver and kidney function, hypertension, protein in the urine, etc., the drug dose will be halved. Suppose they continue to be unable to tolerate the treatment. In that case, the drug should be discontinued, symptomatic treatment should be given, and the treatment should be continued until the toxic and side effects have significantly diminished or disappeared. Group B was administered sorafenib (Bayer Pharma AG; H20130137; 200 mg) orally, 400 mg/time, twice daily (specification: 200 mg).

### 2.4 Observation indicators

Before and three months after treatment, electrocardiogram and laboratory index examinations were performed on the patients. Patients’ 6ml of fasting venous blood was collected and divided between two tubes. A. One tube was centrifuged at 3000r/min for 10 minutes, with a centrifugal radius of 10cm, before being placed in a -80°C for cold storage inspection. Chemiluminescence was used to detect alpha-fetoprotein (AFP), carcinoembryonic antigen (CEA), carbohydrate antigen 199 (CA199), and hypoxia-inducible factor (HIF-1). In this study, vascular endothelial growth factor (VEGF), osteopontin (OPN), epidermal growth factor 7 (EGF7) and other indicators were detected by enzyme-linked immunosorbent assay (ELISA). [Alpha-fetoprotein (AFP): ELISA double antibody sandwich method was used to add samples to the micropores of polystyrene reaction plate coated with anti-AFP antibody. Then, enzyme labeled anti-AFP antibody was added, enzyme substrate was added for color development, reaction was terminated with termination solution, absorbance value was determined, optical density was determined, standard curve was checked, and AFP content in the sample to be measured was calculated. Carcinoembryonic antigen (CEA): ELISA double antibody sandwich normal anti-CEA antibody coated polystyrene reaction plate micropores to add the sample to be tested, then add enzyme labeled anti-CEA antibody, add enzyme substrate color, stop the reaction with termination solution, determine the absorbance value, determine the optical density, check the standard curve, calculate the CEA content in the sample to be tested. Carbohydrate antigen 199 (CA199): Double antibody sandwich method was used. Step 1: Specimen, biotinized anti-CA199 monoclonal antibody and nail (Ru) -labeled anti-CA199 monoclonal antibody are mixed to form sandwich complex. Step 2: Add streptavidin coated particles and allow the resultant complex to bind to the particles through the reaction between biotin and streptavidin. Step 3: The reaction mixed liquid is sucked into the measuring tank, the particles are adsorbed to the electrode through the magnet, the unbonded material is washed away by the cleaning liquid, the electrode is applied voltage to produce chemiluminescence, and the photomultiplier tube is used for measurement. The test result is automatically checked by the machine from the standard curve. This curve is corrected by the instrument with a 2-point calibration, which is obtained from the original standard curve scanned into the instrument from the reagent bar code. Hypoxia-inducible factor (HIF-1): The hypoxia-Inducible factor (HIF-1) was determined by human Hypoxia inducible factor 1a(HIF-1a) enzyme-linked immunosorbent assay (elisa) kit. Enzyme-linked immunosorbent assay (ELISA): Double antibody sandwich ELISA involves the coating of the first antibody (the capture antibody) on a solid vector. After isolation, the antigen to be tested is added, and after incubation, the second antibody (detection antibody) is added. Trapping and detecting antibodies can be two monoclonal antibodies targeting different epitopes, or one monoclonal antibody and one polyclonal antibody targeting the same antigen, but the detection of antibodies requires enzyme labeling.] B. CD4+/CD8+ was evaluated using a NovoCyte D2061R flow cytometer to detect the amounts of CD3+, CD4+, and CD8+ markers of T cell subsets. Aspartate aminotransferase (AST) index was determined using a Roche c701 automatic biochemical analyzer. (2) Record progression-free survival (PFS): From the date of the first dose until disease progression or death from any cause; median overall survival (MS): From the date of the first dose until death from any cause. Date of death or last follow-up for the patient. (3) Safety: According to the American Cancer Institute Adverse Event Terminology Standard (9), the toxic and side effects were graded from 1 to 5, and gastrointestinal reactions (nausea, vomiting, diarrhoea), secondary hypertension, hand-foot syndrome, oral mucositis, and thrombocytopenia were recorded.

The article "A novel therapeutic strategy of combined camrelizumab and apatinib for the treatment of advanced hepatocellular carcinoma" was retracted in 2024. Reasons: compromised peer review; concerns about the results or conclusions; concerns about the peer review; concerns about a third party's involvement.

### 2.5 Efficacy criteria

After 3 months of treatment, the curative effect was evaluated using the relevant criteria from the Expert Consensus on Standardized Diagnosis and Treatment of Primary Liver Cancer (10) and the Modified Response Evaluation Criteria in Solid Tumors (mRECIST) (11). A. Complete remission (CR): The patient’s lesions disappeared on the enhanced imaging in the arterial phase; B. Partial remission (PR): The total of the target lesion diameters (enhanced arterial phase) decreased by at least 30 percent relative to the diameters before treatment; C. Stable disease (SD): The total diameters of the target lesions decreased by less than 30 per cent or increased by less than 20 per cent compared to those before treatment; D. Disease progression (PD): The sum of the diameters of target lesions increased by 20% or more compared with that before treatment, or new lesions appeared.

Objective response rate (ORR) calculation formula: [(CR cases + PR cases)/total cases] × 100.00%; Disease control rate (DCR) calculation formula: [(CR cases + PR cases + SD cases)/total number of cases]×100.00%.

### 2.6 Statistical methods

SPSS 24.0 statistical software was used to analyze and process the enumeration and measurement data in this study, which conformed to normal distribution and uniformity of variance. The measurement data were represented by the median (interquartile range) “M (QR)”, and the Mann-Whitney U test was used to compare the groups. As the test level, the two-sided α =0.05 was used, and the difference was statistically significant when P<0.05.

## 3 Results

### 3.1 Comparison of clinical efficacy between the two groups

-.2As indicated in **Table S2**, the ORR of group A was significantly greater than that of group B after treatment B (χ2 = 4.995, P=0.025), and the DCR of group A was significantly more than that of group B (χ2 = 30.490, P=0.048).

### 3.2 Comparison of tumor markers between the two groups

Before treatment, there was no significant difference between the AFP, CA199, CEA, and HIF-1 indexes of the two groups of patients (P>0.05). After treatment, the tumor markers decreased in both groups. AFP, CA199, CEA, and HIF-1 indexes in group A decreased significantly (P<0.01) compared to group B after treatment. There were significant differences between the groups (P<0.05) as shown in **Table S3**.

The article "A novel therapeutic strategy of combined camrelizumab and apatinib for the treatment of advanced hepatocellular carcinoma" was retracted in 2024. Reasons: compromised peer review; concerns about the results or conclusions; concerns about the peer review; concerns about a third party's involvement.

### 3.3 Comparison of immune function between the two groups

Comparing the two groups’ CD3+, CD4+, CD8+, and CD4+/CD8+ indexes before treatment revealed no significant difference (P>0.05). After treatment, CD3+, CD4+, CD8+, and CD4+/CD8+ indexes in group A increased, while CD8+ indexes decreased (P<0.05), and the improvement of immune function indexes in group A was better than that in group B (P<0.05) as shown in **Table 1** and **Figure 1**.

**Table 1:** Comparison of immune function indexes between the two groups before and after treatment ( $\bar{x}\;\pm \;s$ ).

Group	Number of cases	Time	CD3+(%)	CD4+(%)	CD8+(%)	CD4+/CD8+
A	42	Before Treatment	54.69 ± 5.51	36.14 ± 3.63	27.63 ± 3.10	1.32 ± 0.34
		After Treatment	57.62 ± 6.26	38.32 ± 3.82	24.54 ± 2.29	1.62 ± 0.38
		*t*	2.277	2.681	5.196	3.813
		*P*	0.025	0.009	<0.01	<0.01
B	41	Before Treatment	54.48 ± 5.44	36.05 ± 3.61	27.56 ± 3.07	1.39 ± 0.37
		After Treatment	52.62 ± 5.37	35.68 ± 3.54	27.36 ± 2.83	1.30 ± 0.24
		*T*	1.558	0.469	0.307	1.307
		*P*	0.123	0.641	0.760	0.195

**Figure 1:** Bar graph of comparison of immune function indexes between the two groups before and after treatment $\left(\bar{x}\right)$ .

### 3.4 Comparison of serum indexes between the two groups

Before treatment, there was no significant difference in the two groups VEGF, OPN, Egflt, and AST indexes (P>0.05). After treatment, the VEGF, OPN, Egflt, and AST indexes decreased significantly (P<0.05). Compared to group B, the VEGF, OPN, Egflt, and AST indexes of group A were reduced, with significant differences (P<0.05), as shown in **Table 2** and **Figure 2**.

**Table 2:** Comparison of VEGF, OPN, Egflt and AST between the two groups before and after treatment ( $\bar{x}\;\pm \;s$ ).

Group	Number of cases	Time		VEGF (ng/mL)	OPN (μg/L)	Egflt (μg/L)	AST (U/L)
A	42	Before Treatment		153.87 ± 8.96	27.61 ± 4.02	3141.15 ± 246.84	62.47 ± 7.16
		After Treatment		73.55 ± 4.32^*^	16.38 ± 2.43^*^	1362.42 ± 103.42^*^	31.62 ± 3.07^*^
		t		52.330	15.494	43.073	25.664
		P		<0.01	<0.01	<0.01	<0.01
B	41	Before Treatment		153.76 ± 8.82	27.69 ± 4.25	3140.89 ± 246.76	62.40 ± 7.09
		After Treatment		105.16 ± 6.43	20.07 ± 3.13	1863.27 ± 116.57	42.69 ± 3.56
		t		28.512	9.244	29.976	15.908
		*P*		<0.01	<0.01	<0.01	<0.01

*Compared with group B after treatment, *P<0.05.

The article "A novel therapeutic strategy of combined camrelizumab and apatinib for the treatment of advanced hepatocellular carcinoma" was retracted in 2024. Reasons: compromised peer review; concerns about the results or conclusions; concerns about the peer review; concerns about a third party's involvement.

**Figure 2:** Bar graph of comparison of tumor markers before and after treatment between the two groups $\left(\bar{x}\right)$ .

### 3.5 Comparison of survival time between the two groups

The patients were followed for 24 months after treatment. As indicated in **Table 3**, the PFS and MS of group A were significantly longer than those of group B, with a significant difference (P<0.05).

**Table 3:** Comparison of survival time between two groups ( $\bar{x}\;\pm \;s$ , months).

Groups	Number of cases	PFS	MS
A	42	8.14 ± 2.05	13.34 ± 2.62
B	41	5.34 ± 1.28	9.24 ± 2.37
*T* value		7.443	7.471
*P* value		0.000	0.000

### 3.6 Safety

The toxic and side effects in both groups of patients were mild, and the patients could tolerate them. After symptomatic treatment, the symptoms subsided or improved. **Table 4** shows no significant difference in the side effects of groups A and B (P>0.05).

**Table 4:** Comparison of toxic and side effects between the two groups (example, %).

Groups	Number of cases	Gastrointestinal reactions	Secondary hypertension	Oral mucositis	Thrombocytopenia	Hand-foot syndrome
A	42	22(52.38)	16(38.10)	6(14.29)	2(4.76)	9(21.43)
B	41	18(43.90)	15(36.59)	4(9.76)	1(2.44)	8(19.51)
*x* ^2^		1.440	0.049	0.970	0.776	0.113
*P*		0.230	0.825	0.325	0.379	0.737

## 4 Discussion

HCC is a type of malignant tumor with a high clinical incidence and serious consequences for life and health. According to available data, approximately 393,000 new HCC patients are diagnosed yearly (12). Although radical resection is the treatment of choice for HCC, most patients are diagnosed in the middle and late stages, with a low surgical resection rate and a poor prognosis. Local treatments like radiofrequency ablation and transcatheter arterial chemoembolization (TACE) can only be used to relieve symptoms and improve life quality. Therefore, clinical research actively investigates innovative and effective therapy options for HCC patients. In recent years, molecular targeted therapy and immunotherapy have made significant progress, and the prognosis for some HCC patients has improved significantly. Due to HCC’s high malignancy and poor prognosis, the efficacy of single-drug therapy is limited. Combination therapy is expected to boost the efficacy even further and prolong survival.

To suppress tumor growth, development, and metastasis, molecular targeted therapy targets the over-expressed molecules of tumor cells, and the application of targeted blockers is regulated by the targeted molecules, which are closely linked signal transduction pathways. Sorafenib is a multi-kinase inhibitor with two distinct antitumor effects by inhibiting the MEK, Raf, and ERK signalling pathways. Secondly, it also inhibits the vascular endothelial growth factor receptor 2 (VEGFR-2), c-Kit and platelet-derived growth factor receptor (PDGFR), thus, inhibiting the angiogenesis and tumor cell proliferation indirectly. Studies have demonstrated that sorafenib can halt the progression of advanced HCC tumors and prolong survival. Still, its multitarget mode of action also indicates that it has a wide range of undesirable side effects, and the drug’s high cost limits its clinical application (13). As a result, the clinical trial began investigating more effective combination therapy. Apatinib is a small-molecule anti-angiogenic drug that efficiently inhibits the activity of VEGFR-2 tyrosine kinase, blocks signal transduction mediated by VEGF binding to the receptor, and inhibits tumor vascular endothelial cell migration and proliferation leading to strong anti-tumor impact. Apatinib has a high affinity, and its affinity for VEGFR-2 is 10 times greater than sorafenib, which is more favourable to liver cancer patients (14). Luo Qian (15) emphasized that, as an inflammation-related malignant tumor, the immunosuppressive microenvironment of HCC can develop immunological tolerance *via* many mechanisms. Combining immunotherapy and molecularly targeted therapy has become a new research hotspot to trigger a tumour-specific immune response. Inhibitors of PD-1/PD-L1 are developing immunotherapy that can effectively block the PD-1/PD-L1 signalling pathway, ameliorate the tumor immune microenvironment, restore the anti-tumor activity of immune cells, and enhance endogenous anti-tumor activity. Camrelizumab is a PD-1 blocker that can bind to the PD-1 receptor and disrupt the PD-1/PD-L1 therapeutic pathway. Modern pharmacological studies have demonstrated that camrelizumab may bind to the T-cell-expressed PD-1 receptor and the ligands PD-L1 and PD-L2, which suppress the proliferation of T cells and the production of cytokines and have an effective antitumor effect. Based on arterial chemoembolization combined with camrelizumab in the treatment of advanced HCC, Yang Weihao et al. (16) found that the tumor control rate was higher and survival time was improved. TACE combined with camrelizumab is effective in treating advanced liver cancer, with DCRs of 86.6% at 1 month and 77.4% at 3 months (17). The combination of camrelizumab and HCC is advantageous for patients with liver cancer and HCC. In this study, the ORR and DCR of group A were significantly higher than those of group B, supporting the efficacy of the combination of apatinib and camrelizumab in treating patients with liver cancer and HCC. And combination of apatinib and camrelizumab has a significant improvement compared to Apatinib alone for hepatocellular carcinoma (18). This saves costs to some extent. From the mechanism analysis, carrellizumab can bind to the PD-1 receptor expressed by T cells, and play a certain inhibitory role in the production of cytokines and T cell proliferation factors (19). The clinical efficacy of advanced HCC is better than that of sorafenib alone, as the combined therapy can exert a synergistic effect *via* numerous pharmacological mechanisms, increasing the short-term efficacy.

The article "A novel therapeutic strategy of combined camrelizumab and apatinib for the treatment of advanced hepatocellular carcinoma" was retracted in 2024. Reasons: compromised peer review; concerns about the results or conclusions; concerns about the peer review; concerns about a third party's involvement.

HCC is a malignant tumor with a poor prognosis and a significant risk of metastasis. In clinical practice, tumor marker detection is frequently used for tumor diagnosis, disease dynamics, and prognosis monitoring. AFP is a glycoprotein that is overexpressed in various cancers, including pancreatic cancer, lung cancer, gastric cancer, and HCC. AFP promotes the progression of HCC by inducing T lymphocyte apoptosis through its immunosuppressive effect. According to studies, 27% of patients with benign liver disease have high AFP expression, 40% of patients with liver cancer have no obvious increase in serum AFP, and some patients with early HCC have normal AFP levels (20). The sensitivity of detecting AFP alone is low. CA199 and CEA are common tumor markers that are found in lung cancer, esophageal cancer, hepatocellular carcinoma, and other types of cancer. HIF-1 is a hypoxia-dependent protein that can mediate VEGF and angiopoietin (Ang) 2 signalling, induce tumor angiogenesis, and play a role in tumor cell infiltration and metastasis. According to the findings of Zhang Hui et al. (21), AFP, CA199, and CEA levels in HCC patients were significantly higher than in the benign liver disease group and healthy subjects. In contrast, CA199 and CEA levels in the benign liver disease group were significantly higher than those in healthy subjects. Consequently, the concurrent detection of AFP, CA199, CEA, and HIF-1 can dynamically grasp the condition of HCC and evaluate prognosis. In this study, the AFP, CA199, CEA and HIF-1 indexes of the two groups decreased after treatment, and the AFP, CA199, CEA and HIF-1 indexes of group A were significantly lower than those of group B, suggesting that apatinib combined with camrelizumab Antibiotics can further reduce the level of serum tumor markers in HCC patients. The reason is that camrelizumab can block the immunosuppressive state of T lymphocytes mediated by the PD-1 pathway, promote the activation of T lymphocytes, and rebuild the body’s immune function, thereby reducing the level of tumor markers. After treatment in group A, CD3+, CD4+, CD4+/CD8+ increased, while CD8+ indexes decreased. CD3+, CD4+, CD4+/CD8+ after treatment in group A were significantly higher than those in group B. In contrast, CD8+ in group B was significantly lower than that in group B after treatment. There was no significant difference in T lymphocyte subset indicators between before and after treatment, indicating that the combination of apatinib and camrelizumab has significant benefits for enhancing the immune function of HCC patients. HCC is a typical highly vascularized tumor; its growth, invasion, and metastasis (22) are inherently associated to angiogenesis. VEGF is the most specific and potent pro-angiogenic factor, and it plays a significant role in HCC growth, invasion, and metastasis, in addition to being associated with prognosis. OPN is a widely distributed phosphorylated glycoprotein with diversified biological functions. It is secreted and widely distributed in human tissues. The protein can mediate immune responses, and intercellular adhesion, participate in cell signalling, etc promotes the growth and invasion of tumor cells. Studies by Zheng Yan et al. (23) indicate that VEGF and OPN are abnormally elevated in liver cancer patients and are higher in tumor thrombus formation, metastasis, and poorly differentiated tumors. Egfl7 is a secreted protein that enhances vascular endothelium’s and fibroblasts’ migratory ability and promotes tumor invasion and metastasis by activating chemotactic signals. Sun Xiaoying (24) demonstrated that the blood Egfl7 level in HCC patients was significantly higher than in healthy volunteers, and its level was significantly associated with tumor size, confirming its role in the occurrence and progression of HCC. AST is a biochemical marker for evaluating the liver function, and its serum concentration is elevated in the presence of serious liver lesions or necrosis. Huang Jianxiang found that in HCC patients with microvascular invasion, combined camrelizumab therapy based on TACE treatment, VEGF, OPN, and Egfl7 levels were substantially decreased at 1 month and 3 months after surgery compared to before treatment and the degree of reduction was higher than in patients treated with TACE alone, and the quality of life was higher in patients treated with combination therapy. As a result, HCC patients may benefit from the downregulation of serum VEGF, OPN, and Egfl7 indexes (25). In this study, the VEGF, OPN, Egfl7, and AST indexes decreased in both groups after treatment, with group A decreasing more significantly than group B, implying that apatinib combined with camrelizumab in the treatment of advanced HCC can further improve the outcomes. It can lower serum levels of VEGF, OPN, and Egfl7 in patients and prevent liver damage, which is one of the key reasons for the large reduction in tumor marker levels in HCC patients treated with combination therapy and the further improvement of the curative effect. This study had a median follow-up period of 13 months. PFS and MS were significantly longer in group A than in group B, but neither group experienced severe toxic or side effects that could not be alleviated or avoided by symptomatic treatment. However, there was no significant difference, suggesting that the combination of apatinib and camrelizumab can prolong the survival of HCC patients without significantly increasing toxicity and side effects, demonstrating its efficacy and safety.

The article "A novel therapeutic strategy of combined camrelizumab and apatinib for the treatment of advanced hepatocellular carcinoma" was retracted in 2024. Reasons: compromised peer review; concerns about the results or conclusions; concerns about the peer review; concerns about a third party's involvement.

In conclusion, the clinical application of apatinib combined with camrelizumab in the treatment of patients with advanced HCC has a significant curative effect, good tolerance, and can prolong the survival of patients. Its pharmacological mechanism may be associated with the reduction of levels of tumor markers and the regulation of immune function, as well as the down-regulation of levels of VEGF, OPN, and Egfl7.

## Data availability statement

The original contributions presented in the study are included in the article/**Supplementary Material**. Further inquiries can be directed to the corresponding authors.

## Author contributions

QY and GL have contributed equally to this work and share first authorship. CS and SZ contributed equally to this work as corresponding authors. All authors contributed to the article and approved the submitted version.
